# Therapeutic targets and limits of minocycline neuroprotection in experimental ischemic stroke

**DOI:** 10.1186/1471-2202-10-126

**Published:** 2009-10-06

**Authors:** Noriyuki Matsukawa, Takao Yasuhara, Koichi Hara, Lin Xu, Mina Maki, Guolong Yu, Yuji Kaneko, Kosei Ojika, David C Hess, Cesar V Borlongan

**Affiliations:** 1 Department of Neurology, Medical College of Georgia, Augusta, GA 30912, USA; 2 Department of Neurology and Neuroscience, Nagoya City University Graduate School of Medical Sciences, Nagoya, 467-8601, Japan; 3 Research and Affiliations Service Line, Augusta VAMC, Augusta, GA 30912, USA

## Abstract

**Background:**

Minocycline, a second-generation tetracycline with anti-inflammatory and anti-apoptotic properties, has been shown to promote therapeutic benefits in experimental stroke. However, equally compelling evidence demonstrates that the drug exerts variable and even detrimental effects in many neurological disease models. Assessment of the mechanism underlying minocycline neuroprotection should clarify the drug's clinical value in acute stroke setting.

**Results:**

Here, we demonstrate that minocycline attenuates both *in vitro *(oxygen glucose deprivation) and *in vivo *(middle cerebral artery occlusion) experimentally induced ischemic deficits by direct inhibition of apoptotic-like neuronal cell death involving the anti-apoptotic Bcl-2/cytochrome c pathway. Such anti-apoptotic effect of minocycline is seen in neurons, but not apparent in astrocytes. Our data further indicate that the neuroprotection is dose-dependent, in that only low dose minocycline inhibits neuronal cell death cascades at the acute stroke phase, whereas the high dose exacerbates the ischemic injury.

**Conclusion:**

The present study advises our community to proceed with caution to use the minimally invasive intravenous delivery of low dose minocycline in order to afford neuroprotection that is safe for stroke.

## Background

Cerebral ischemia triggers a cascade of pathophysiological events including excitotoxicity, ionic imbalance, oxidative and nitrosative stresses and apoptotic-like cell death mechanisms [1-8]. To date, the thrombolytic agent tPA is the only effective drug for acute ischemic stroke; however, only about 2% of ischemic stroke patients benefit from this treatment due to its limited therapeutic window [9]. There is a desperate need to develop additional neuroprotective strategies [10-12]. Minocycline is a promising neuroprotectant because if is safe, easily penetrates the CNS, and effective in various models of acute neurological injury.

Cell death associated with the initial blood flow interruption and the immediately ensuing excitotoxity is abrupt, while inflammation occurs over a long period of time from stroke onset. Accordingly, anti-inflammatory treatment is likely to extend the therapeutic window allowing improved intervention in stroke. Indeed, minocycline, a common tetracycline antibiotic, has been demonstrated to provide neuroprotection against ischemic brain via the inhibition of the inflammatory cascade [13-15]. Accumulating evidence indicates that minocycline exerts neuroprotective effects in neurodegenerative disease models, such as Parkinson's disease, Alzheimer's disease, multiple sclerosis, spinal cord injury, and Huntington's disease [16-24]. Depending on the experimental injury paradigm [19], minocycline may promote neuroprotection through inhibition of microglial activation via p38 against NMDA excitotoxicity [25] ischemic injury [26], NO [27], glutamate [28] and MPTP excitotoxicity [17], or through suppression of apoptotic cell death via Bcl-2/cytochrome c against ischemia in kidney cells [29], heat stress in testes [30], and NO excitotoxicity in vascular smooth muscle [31], spinal cord injury [32] and ALS [33]. In animal models of stroke, minocycline has been reported to reduce infarct volume and to attenuate behavioral deficits [34-37] via the inhibition of microglial activity [13-15]. Overall, the commonly postulated pathway of minocycline neuroprotection in stroke focuses on the modulation of microglial activity. However, because the acute stage of stroke involves abrupt neuronal injury prior to inflammatory reaction, the demonstration of minocycline protection against the primary ischemic cell death would be of high therapeutic interest. Moreover, whereas the inhibition of microglial activity by minocycline against ischemia has been shown to highly correlate with the dose [15,34-40], the possibility of neurotoxicity of minocycline at higher doses has only been recently recognized [41,42].

In this study, we examined direct protective effects of minocycline on neurons and astrocytes, and also determined minocycline's toxicity profile in both *in vitro *and *in vivo *models of stroke. The overarching theme is to provide guidance on advancing minocycline therapy to the clinic by assuring the safety of the drug and further understanding the feasibility of a direct neuroprotective treatment in view of the acute cell death associated with ischemic stroke.

## Results

### Minocycline improves cell viability of neurons, but not astrocytes

Based on ATP activities (MTT assay), minocycline, at low doses, maintained cell viability of primary cultured neurons exposed to OGD (0.001 μM: 85.9 ± 13.1%, 0.01 μM: 94.4 ± 7.2%, 0.1 μM: 90.4 ± 13.0%, 1 μM: 88.2 ± 13.8%; values hereon are expressed relative to non-OGD exposed group) compared to vehicle treated group (0 μM: 67.1 ± 10.3%), but was toxic at high dose (100 μM: 55.1 ± 8.4%) (F_7,32 _= 14.775, p < 0.0001) (Figure 1A). In contrast, minocycline, at all doses, did not exert neuroprotective effects on primary cultured astrocytes, and additionally was toxic at high dose (100 μM: 49.5 ± 5.0%) compared to vehicle-treated group (0 μM: 72.6 ± 4.3%) (F_7,32 _= 16.255, p < 0.0001) (Figure 1B). Similarly, Trypan blue results mimicked those of MMT data, in that cell viability of neurons, but not astrocytes, was maintained by low doses of minocycline (neurons: 0.01 μM: 66.6 ± 10.9%, 0.1 μM: 87.6 ± 2.9%, 1 μM: 77.3 ± 8.2%), while high dose minocycline was toxic to both neurons and astrocytes (neurons: 100 μM: 10.5 ± 4.7%; astrocytes: 100 μM: 43.3 ± 7.7%) compared to vehicle-treated group (neurons: 0 μM: 56.3 ± 6.9%, F_7,32 _= 57.300, p < 0.0001, astrocytes: 0 μM: 43.3 ± 7.7%, F_7,32 _= 27.989, p < 0.0001) (Figure 1C-L).

**Figure 1:** **ATP activity and trypan blue assay in cultured neurons and astrocytes**. ATP activity was measured to reveal cell viability with varying concentrations of minocycline or vehicle. OGD condition reduced ATP activity of cultured neurons to 40% of non-OGD control group (A). Low doses of minocycline (0.001 to 10 μM) preserved cell viability of neurons (A), but not astrocytes (B). In contrast, high dose of minocycline (100 μM) displayed toxicity to both neurons and astrocytes (A, B). In parallel with ATP assay, Trypan blue assay revealed that low doses of minocycline (0.001-10 μM) exerted neuroprotective effects on cultured neurons, but not astrocytes (C-G: neurons, H-L: astrocytes, C, H: non-OGD control, D, I: 0 μM, E, J: 1 μM, F, K: 100 μM of minocycline). High dose of minocycline (100 μM) displayed toxicity for both neurons and astrocytes. Data are shown as mean values ± SEM (*p < 0.05 increase and **p < 0.05 decrease vs. vehicle-treated cultured neurons or astrocytes; A, G: neurons, B, L: astrocytes). Scale bar: 25 μm.

### Minocycline alters OGD-induced apoptotic cell death

The cell death of neurons and astrocytes under OGD condition represents apoptotic-like cell damage as revealed by caspase 3/7 assay (neurons: 29927.5 ± 6365.4/well; astrocytes: 17758.5 ± 5.78.9 well) (Figure 2A, B) and TUNEL assay (neurons: 189.6 ± 18.8 cells/0.2 mm^2^; astrocytes: 60.7 ± 2.8 cells/0.2 mm^2^) (Figure 2I, J). Compared to normal, non-OGD conditions, OGD increased caspase activity levels by about 1.5-fold. Treatment with low dose minocycline prevented such apoptotic-like cell death in neurons characterized by reduced caspase 3/7 activity (neurons: 16675.8 ± 2474.2/well) (F_2,12 _= 19.611; p = 0.0002) (Figure 2A) and decreased TUNEL positive cells (55.0 ± 13.2 cells/0.2 mm^2^) (F_2,12 _= 13.26; p < 0.001) (Figure 2C-E, I). However, protective effects of low dose minocycline were not detected in astrocytes (caspase: 22705.9 ± 2268.0/well, TUNEL: 83.7 ± 4.544 cells/0.2 mm^2^) (Figure 2B, F-H, J). Moreover, minocycline, at a high dose, worsened apoptotic-like cell death in both neurons (caspase: 35600.0 ± 3450.4/well), (TUNEL: 234.0 ± 33.7 cells/well) and astrocytes (caspase: 30708.0 ± 2901.3/well) (F_2,12 _= 9.831; p = 0.0030), (TUNEL: 75.8 ± 10.5 cells/0.2 mm^2^) (F_2,12 _= 4.76; p < 0.01) (Figure 2A, B, I, J).

**Figure 2:** **Caspase3/7 activity and tunel staining in cultured neurons and astrocytes**. Low dose minocycline (1 μM) reduced caspase3/7 activity of neurons (A), but not of astrocytes (B). In contrast, high dose minocycline (100 μM) displayed no suppressive effects on caspase 3/7 activity of neurons and increased that of astrocytes (A, B). Similarly, low dose minocycline reduced, whereas high dose minocycline increased the number of TUNEL positive neurons compared to vehicle-treated cultured neurons (OGD-exposed neurons treated with 0, 1 and 100 μM of minocycline; panels C, D and E, respectively). On the other hand, minocycline at all doses did not reduce the number of TUNEL positive astrocytes (OGD-exposed astrocytes treated with 0, 1 and 100 μM of minocycline; panels F, G and H, respectively). Data are shown as mean values ± SEM (*p < 0.05. A, I: neurons, B, J: astrocytes). Scale bar: 50 μm.

Under OGD condition, increased Bcl-2 expression was induced by low dose minocycline in cultured neurons (0 μM: 1.25 ± 0.48, 1 μM: 18.9 ± 2.16 cells/0.05 mm^2^), but not at a high dose (100 μM: 2.21 ± 1.10 cells/0.05 mm^2^) (F_2,12 _= 15.288; p = 0.004) (Figure 3A-D, H). In contrast, Bcl-2 expression was not altered by minocycline at all doses in astrocytes (0 μM: 3.33 ± 2.11, 1 μM: 1.67 ± 1.67, 100 μM: 0.0 ± 0.0 cells/0.05 mm^2^) (Figure 3A, E-G, I). In parallel, the OGD-induced release of cytochrome c from mitochondria into cytosol was prevented by minocycline at a low dose in neurons.

**Figure 3:** **Bcl-2 expression and cytochrome c release in cultured neurons and astrocytes**. Western blotting revealed that low dose minocycline upregulated Bcl-2 expression of neurons (A: lysates from 0, 1 and 100 μM of minocycline-treated neurons correspond to lanes 1, 2, and 3, respectively) with subsequent inhibition cytochrome c release from mitochondria to cytosol (B: lysates from 0, 1 and 100 μM of minocycline-treated neurons correspond to lanes 7, 8, and 9, respectively). In contrast, minocycline at all doses did not upregulate Bcl-2 expression in astrocytes (A: lysates from 0, 1 and 100 μM of minocycline-treated astrocytes correspond to lanes 4, 5, and 6, respectively). Immunocytochemical analysis revealed that minocycline low dose (D: 1 μM) significantly increased the number of Bcl-2 positive neurons compared to vehicle-treated (C: 0 μM) or high dose-treated neurons (E: 100 μM). In contrast, minocycline at all doses did not alter the number of Bcl-2 positive astrocytes (F: 0 μM, G: 1 μM and H: 100 μM). Quantitative analyses of Bcl-2 positive cells are shown in panels I and J. Data represent mean values ± SEM (* p < 0.05. I: neurons, J: astrocytes). Scale bar: 25 μm.

### Minocycline ameliorates stroke-induced behavioral deficits

At three days post-stroke, the typical motor and neurological dysfunctions produced by MCAo were significantly blocked by minocycline when intravenously administrated at a low dose (20 mg/kg) starting at 60 minutes after reperfusion, as revealed by EBST (0 mg/kg: 88 ± 12.5%, 20 mg/kg: 68.3 ± 15%) (F_2,27 _= 10.439; p = 0.0004) (Figure 4A) and Bederson test (0 mg: 1.67 ± 0.14, 20 mg/kg: 1.16 ± 0.36) (Kruskal-Wallis H value = 19.2, df = 2, p < 0.0001) (Figure 4B). In contrast, MCAo stroke animals treated with high dose minocycline (100 mg/kg) displayed neurological deficits (Bederson: 2.15 ± 0.38) that were significantly worse and their motor deficits were slightly exacerbated (EBST: 89 ± 13%; though not significant difference) compared to stroke animals that received vehicle alone. In addition, these stroke animals treated with high dose minocycline performed significantly worse in both behavioral tests than those that received the low dose minocycline (p's < 0.05).

**Figure 4:** **Motor and neurological performance of stroke rats**. Both motor and neurological dysfunctions were significantly ameliorated by low dose minocycline (20 mg/kg, i.v.), as revealed by elevated body swing test (EBST; A) and Bederson test (B). In contrast, high dose minocycline (100 mg/kg, i.v.) significantly exacerbated neurological deficits and slightly worsened motor deficits. Data are shown as the mean values ± SEM (*p < 0.05).

### Minocycline reduces cerebral infarcts

Following behavioral testing at three days post-stroke, TTC staining revealed that the infarct volume was significantly reduced by low dose minocycline (80.1 ± 41.7 mm^3^) relative to vehicle-treated stroke group (138.5 ± 48.8 mm^3^) (F_2,27 _= 9.552; p = 0.0007) (Figure 5A, B, D). In particular, the stroke damage within the striatum was significantly smaller in low dose minocycline-treated stroke animals than vehicle-treated stroke animals. In contrast, the infarct volume in high dose minocycline-treated stroke group was significantly larger than those of vehicle-treated stroke group (180.47 ± 56.1 mm^3^) (Figure 5A, C, D). Indeed, in some high dose minocycline-treated stroke animals, cerebral infarcts were observed even in the hemisphere contralateral to the MCAo side. Posthoc analyses of hemorrhage revealed 20% incidence with an average size of 12 mm^2^, which did significantly differ across treatment groups. Similarly, measurements of edema found no significant differences across groups (although there was a slight reduction in the low dose minocycline group compared to vehicle group), indicating that our analysis of neuronal cell loss (see below) was not affected by edema formation.

**Figure 5:** **Cerebral infarct analysis of stroke brains**. TTC staining revealed that low dose minocycline (20 mg/kg; B) significantly reduced cerebral infarct volumes compared to the vehicle group (A). In particular, the striatal infarct volumes in the low dose group were significantly smaller than the vehicle group. In contrast, high dose minocycline (100 mg/kg; C) significantly increased the infarct volumes compared to those in the vehicle group. Quantitative analyses are shown in panel D. Data represent mean values ± SEM (*p < 0.05).

### Minocycline abrogates MCAo-mediated apoptotic cell death

A new set of animals (n = 18) underwent MCAo, randomly assigned to similar minocycline treatment as described above, and euthanized at three days post-stroke for immunohistochemical analyses of apoptotic cell death. Results revealed that Bcl-2 immunoreactivity was significantly increased in the brains of stroke animals that were treated with low dose minocycline, especially within the striatum ipsilateral to the occluded MCA (20 mg/kg: 9.83 ± 1.50 density/0.05 mm^2^) relative to vehicle-treated stroke animals (0.235 ± 0.112 cells/0.05 mm^2^) (F_2,15 _= 37.151; p < 0.0001) (Figure 6A, B, D). In contrast, Bcl-2 immunoreactivity in the same striatal area of high dose minocycline-treated stroke animals was not significantly differrent from vehicle-treated stroke animals (100 mg/kg: 1.14 ± 0.22 density/0.05 mm^2^) (Figure 6A, C, D). To clarify which cell type expresses Bcl-2, we examined double-labeling of Bcl-2 with MAP2 or GFAP by immunohistochemistry in ischemic striatal peri-infact area of each group. Bcl-2 was found co-localized with MAP2 in all groups (Figure 6F-H). In contrast, GFAP positive astrocytes did not express Bcl-2 (Figure 6I-K). These results suggest that low dose minocycline can exert anti-apoptotic effects via Bcl-2 upregulation in ischemic neurons. A few cells in vehicle-treated stroke rats also expressed Bcl-2 and MAP2 double-labeling, indicating that ischemia alone, without any treatment intervention, might slightly induce the expression of Bcl-2 in neurons.

**Figure 6:** **Tunel staining in the ischemic peri-infarct area**. Low dose significantly decreased (B), whereas high dose significantly increased (C) the number of TUNEL positive cells in the ischemic striatal peri-infarct area of minocycline-treated stroke rats compared to the vehicle-treated stroke rats (A). Quantitative analyses of Bcl-2 positive cells are shown in panel D. Data are shown as mean values ± SEM (*p < 0.05). Four representative ischemic striatal peri-infarct areas (+0.2 mm anterior to the bregma), in which TUNEL positive cells were counted (data in panel D), are shown in panel E (square boxes labeled 1-4 correspond to areas 1-4 in panel D). Scale bar: 25 μm.

In addition, whereas TUNEL-positive cells with agglutinated nuclei highly populated the striatal peri-infarct area of high dose minocycline treated or vehicle treated animals, there were significantly fewer TUNEL-positive cells in animals treated with low dose minocycline (F_2,15 _= 35.411; p < 0.0001) (Figure 7A-D). Similar dose dependent anti-apoptotic effects were obtained from Bcl-2 immunohistochemistry, in that low dose minocycline significantly increased the number of Bcl-2 positive cells within the striatal peri-infarct area compared to high dose minocycline or vehicle treatment.

**Figure 7:** **Bcl-2 expression in the ischemic peri-infarct area**. Low dose (B) significantly upregulated, whereas high dose (C) significantly suppressed the Bcl-2 expression in the ischemic peri-infarct area of minocycline-treated rats compared to that in the vehicle-treated rats (A). Quantitative analyses of Bcl-2 positive cells are shown in panel D. Data are shown as mean values ± SEM (*p < 0.05). Two representative ischemic striatal peri-infarct areas (+0.2 mm anterior to the bregma), in which Bcl-2 positive cells were counted (data in panel D), are shown in panel E (square boxes). Co-localization of Bcl-2 and MAP2 was found in ischemic striatal peri-infarct area, suggesting anti-apoptotic effects of minocycline via Bcl-2 upregulation in ischemic neurons (F-H). In contrast, GFAP positive astrocytes did not express Bcl-2 (I-K). Scale bar: 25 μm (A-C), 12.5 μm (F-K); asterisks (*): merged cell; green and red immunofluorescent markers correspond to Bcl-2 and MAP2, respectively.

### Minocycline rescues neurons in the peri-infarct area

To determine the effect of minocycline on neurons *in vivo*, we examined the number of Nissl positive cells in ischemic peri-infarct area on consecutive brain sections. Vehicle-treated MCAo stroke rats exhibited neuronal cell loss in the peri-infarct area (152.0 ± 10.0 cells/0.05 mm^2^) relative to intact brain (303.3 ± 13.9 cells/0.05 mm^2^) (Figure 8A, B, E). Low dose minocycline (228.3 ± 6.9 cells/0.05 mm^2^) revealed significant protective effect relative to vehicle treated group (152.0 ± 10.1 cells/0.05 mm^2^) (F_3,16 _= 4 9.488; p < 0.0001) (Figure 8B, C, E), as well as retained fundamental structure of striatum. In contrast, high dose minocycline (104.3 ± 6.8 cells/0.05 mm^2^) revealed significant neuronal cell loss (104.3 ± 16.4 cells/0.05 mm^2^) relative to vehicle treated group (though no significant difference), in addition to dissolution of fundamental structure of striatum with severe edema (Figure 8B, D, E).

**Figure 8:** **Neuronal survival in the ischemic peri-infarct area**. Neuronal survival in the ischemic striatal peri-infarct area, visualized with cresyl violet stain, was significantly preserved by low dose minocycline (A: intact control, B: vehicle, C: 20 mg/kg, D: 100 mg/kg). In contrast, high dose minocycline resulted in the collapse of fundamental neuroarchitecture of the striatum accompanied by severe edema. Data are shown as mean values ± SEM (*p < 0.05). Scale bar: 25 μm.

## Discussion

The present study demonstrates that minocycline exerted direct protection on neurons, in the absence of astrocyte participation, against ischemic stroke. An equally important finding is that minocycline not only promoted dose-dependent neuroprotective effects, but also induced toxicity at a high dose for both neurons and astrocytes. Both sets of *in vitro *and *in vivo *studies corroborated such neuroprotection and toxicity profile of minocycline. In addition, *in vitro *mechanistic studies revealed that a major therapeutic pathway, by which minocycline prevented the ischemic cell death, is via an anti-apoptotic mechanism. Parallel *in vivo *data showed that low dose, but not high dose, minocycline attenuated stroke-induced behavioral deficits, decreased apoptotic cell death and reduced cerebral infarction. The intravenous route and the post-stroke delivery further advance the utility of minocycline in the clinic.

To date, the primary CNS mechanism implicated in minocycline neuroprotection is the drug's highly potent inhibitory effect on microglial activation, which is achieved by blocking the phosphorylation of p38 and the translocation of 5-Lipoxygenase into the nucleus, thereby preventing the release of cytokines and the induction of inflammation [15,40,43-45]. On the other hand, recent evidence has shown that minocycline in the periphery affords protective effects on kidney cells against ischemia via the apoptotic Bcl-2/cytochrome c pathway [29]. We report here that minocycline also promoted protection against ischemia in the CNS by arresting apoptotic Bcl-2/cytochrome c pathway. In our *in vitro *OGD condition, cultured neurons and astrocytes underwent apoptosis-like cell death as revealed by induction of caspase 3/7 activity and DNA fragmentation (TUNEL positive cells). Treatment with low, but not high dose minocycline abrogated apoptosis characterized by reduced caspase 3/7 activity and decreased number of TUNEL positive cells. Of note, such blockade of OGD-induced apoptosis by low dose minocycline only occurred in cultured neurons and was not evident in cultured astrocytes.

In stroke brains, increased chemokine mRNA expression displays a biphasic profile, being found initially in neurons, then subsequently in astrocytes [46]. Of interest, high levels of chemokines were found in areas of gliosis surrounding recent infarcts [47-49] and correlated with the accumulation of macrophage/microglia in the ischemic lesion, suggesting chemokine's role in the recruitment of inflammatory cells into the brain in response to stroke [49-52]. Based on the above observations, suppressing chemokine elevation during its initial onset in neurons, before astrocytes become involved in this inflammation-ischemia-triggered secondary cell death, may provide better therapeutic outcome than treatment regimen targeting astrocytes. Although in recent years enhancing astrocyte survival has been suggested as an alternative protective approach against ischemic damage [53,54], therapeutic strategies that confer direct neuronal protection are likely to improve clinical prognosis. The present results indicate that minocycline, in addition to its established anti-microglial activity, could directly protect neurons via an anti-apoptotic mechanism.

To further clarify the anti-apoptotic features of minocycline, we examined the alterations in expression of apoptosis-related components, specifically the cell survival-enhancing Bcl-2/cytochrome c pathway. Our results revealed that low dose minocycline protected again neurons, but not astrocytes against OGD by elevating Bcl-2 expression and consequently strengthening the anchor of cytochrome c to the mitochondria. We extend here the participation of Bcl-2/cytochrome c pathway in minocycline's direct protection of OGD-exposed neurons, previously shown in ischemic kidney cells [29].

To reveal the possible toxic side effects of minocycline, we similarly examined cell survival and apoptosis in OGD-exposed cultured neurons and astrocytes treated with high dose (100 μM) minocycline. Minocycline at a high dose was toxic as revealed by markedly reduced cell survival of both OGD-exposed neurons and astrocytes compared to vehicle treated OGD-exposed cells. Moreover, relative to vehicle treated OGD exposed cells, high dose minocycline did not elevate Bcl-2 expression, but increased caspase 3/7 activity, as well as the number of TUNEL positive cells in the ischemic striatum.

In parallel to the toxicity profile of minocycline observed in the *in vitro *OGD condition, high dose minocycline exacerbated both behavioral and histological deficits in stroke animals. In contrast, low dose minocycline increased Bcl-2, but decreased TUNEL positive cells in the ischemic peri-infarct area. Moreover, low dose minocycline-treated animals exhibited a pattern of Bcl-2 expression that was only found in neurons, but not in astrocytes, further supporting the neuroprotective mechanism whereby minocycline exerted anti-apoptotic effects directly on neurons.

In previous reports, therapeutic efficacy in different animal models of neurological disorders was consistently observed when minocycline was administered 3 mg/kg-45 mg/kg either intravenously or intraperitoneally [37-39]. Recent studies have suggested that depending on the animal species (i.e., mice), minocycline may confer neurotoxicity in experimental ischemia [19,38,42] and Parkinson's disease [41]. These reports and the present data, taken together, further clarified the toxicity profile of minocycline highlighting critical factors including type of cell line (for *in vitro *studies), experimental injury paradigm, and dosage, as well as delivery route of minocycline [19,37-39].

The observed dose-dependent protection of neurons over astrocytes by low dose minocycline, and the neurotoxic effects of high dose minocycline provide guidance in designing the clinical protocol for stroke patients. Because astrocytes play a crucial role in blood brain barrier maintenance, a perturbed astrocyte viability, as seen with high dose minocycline, may compromise the barrier that could allow inflammatory cells to penetrate the CNS and exacerbate the stroke deficits. Indeed, most of the animals that received high dose minocycline exhibited severe edema. The establishment of an effective dose range that confers protection on neurons, while not disrupting astrocytes, would perhaps lead to improved therapeutic outcome of minocycline.

Minocycline's inability to protect astrocytes or to increase Bcl-2 expression in these cells *in vitro *seems to be the most original finding of this study. Our approach to use low doses and high doses to show minocycline's protection versus toxicity in the same *in vitro *and *in vivo *stroke models is clinically relevant since the drug is already in clinical trials. At first glance, the choice for the present high doses of minocycline (100 μM or 100 mg/kg) would seem extremely high, considering that in a clinical trial [21] multiple sclerosis patients who received orally 200 mg minocycline daily dose (equals 2.85 mg/kg for 70 kg person, serum levels reach maximum of 4 mg/l = 8 uM) during a 6-month period exhibited no observable significant side effects. However, our recent study clearly demonstrates that a 3 mg/kg intravenous dose of minocycline is required to obtain serum levels in rats similar to that achieved in humans after a standard 200 mg dose [37], suggesting differences in the drug metabolism between rats and humans. Accordingly, the rationale for selecting the present doses of minocycline is based on our studies [37,39] and those of others [13,28,34,55,56] indicating that these doses correspond to the clinically relevant doses of minocycline in stroke rodent models. In addition, we extended the high dose range to reveal the toxicity profile of minocycline. Indeed, a multiple high dose minocycline injection regimen, involving subcutaneous 135 mg/kg over 2 days followed by 68 mg/kg over the succeeding two days, was recently shown to exacerbate the striatal damage produced by hypoxic-ischemic injury in rats [42]. Depending on the dose and route of delivery, discordant results and conclusions accompany the actions of minocycline in various stroke and neurodegeneration models. The present data underscore that the minocycline dose is critical as it might attenuate or worsen the stroke outcome. While many studies have pursued intraperitoneal or subcutaneous injections of high dose minocycline in order to promote neuroprotection, we show here that robust neuroprotective effects in acute stroke can be achieved with intravenous low dose minocycline, thereby circumventing the toxicity now increasingly being recognized with high dose minocycline. This neuroprotective action of low dose minocycline at a clinically suitable dosing regimen advances the entry of this drug for phase I human stroke trials. In view of a recent clinical trial showing that the relatively high dose of 400 mg/day for 9 months minocycline led to an accelerated deterioration in the amyotrophic lateral sclerosis functional rating scale, accompanied by gastrointestinal and neurological adverse events [57], a more careful consideration of minocycline dose is indicated as similarly shown in the present study.

## Conclusion

In conclusion, the safety and therapeutic efficacy of low dose minocycline and its robust neuroprotective effects during acute ischemic stroke make it an appealing drug candidate for stroke therapy. The implication of the present direct minocycline protection of neurons, as opposed to the reported inhibition of microglial activity, can be best appreciated by the fact that stroke triggers abrupt neuronal cell death that would require immediate intervention to rescue ischemic cells. A delay in abrogating the primary stroke-induced cell death could result in "fixed" or devastating histological and functional deficits that will be difficult to repair. Coupled with the ability of minocycline to block the microglial activation occurring at later post-stroke periods, we now provide evidence that minocycline is also able to achieve an expedited direct neuroprotection against ischemia at early time points. To our knowledge, such two-pronged neuroprotective approach targeting both primary and secondary cell death processes associated with stroke has not been shown with monotherapy. Minocycline stands as a multiple site of action therapeutic drug, which clinically should be effective in treating neurological diseases, like stroke, characterized by many facets of cell death cascades.

## Methods

The present experimental research and relevant ethical issues were approved by Veterans Affair Medical Center Institutional Animal Care and Use Committee, and adhered to National Institutes of Health guidelines.

### In vitro study

#### Cell culture

Primary cultures of neurons and astrocytes were derived from the rat (Sprague-Dawley) striatum and maintained in culture following the supplier's protocol (CAMBREX, MD). Briefly, immediately after thawing, cells (4 × 10^4 ^cells/well) were seeded and grown in 96-well plate coated by poly-l lysine in Neurobasal media (GIBCO, CA) containing 2 mM L-glutamine, 2% B27 (GIBCO, CA) and 50 U/ml penicillin and streptomycin for 7-10 days at 37°C in humidified atmosphere containing 5% CO_2_. Purity of the cells were immunocytochemically determined to be > 99% for both neuronal and astrocytic cell population as revealed by DARPP-32 and GFAP immunostaining, respectively. Moreover, we confirmed that these cells were appropriate for the oxygen glucose deprivation (OGD) injury model, where glutamate excitotoxicity plays an important role, as revealed by expression of glutamate receptors (determined immunocytochemically using vesicular glutamate transpoter-1) in 50% of the neuronal and astrocytic cell population.

#### Oxygen-glucose deprivation (OGD)

Cultured cells were exposed to the OGD injury model as described previously [58] with few modifications. Briefly, culture medium was replaced by a glucose-free Earle's balanced salt solution (BSS) with the following composition (116 mM NaCl, 5.4 mM KCl, 0.8 mM MgSO_4_, 1 mM NaH_2_PO_4_, 26.2 mM NaHCO_3_, 0.01 mM glycine, 1.8 mM CaCl_2_, and pH adjusted to 7.4 with or without minocycline. Cultured cells were placed in humidified chamber, then equilibrated with continuous flow of 92% N_2 _and 8% O_2 _gas for 15 minutes. After this equilibrium, the chamber was sealed and placed into the incubator at 37°C for 75 minutes, 2 hours, 4 hours and 12 hours for Western blot, caspase assay, MTT assay and Trypan blue stain, respectively. For Western blot, cells were subsequently exposed to standard medium in 5% CO_2 _incubator for an additional 6 hours to generate apoptosis-related proteins [58].

#### Cell viability

Cell viability was evaluated by ATP activity following the supplier's protocol (Promega, WI) and by Trypan blue (Sigma, MO). Briefly, MTT assay was carried out by adding MTT assay solution immediately after OGD. The intensities of chemiluminescence of ATP activity were measured and calculated by Image station 2000R system (Kodak, NY). In addition, Trypan blue exclusion method was conducted and mean viable cell counts were calculated in three randomly selected areas (0.2 mm^2^) in each well (n = 5 per treatment condition) to reveal the cell viability for each treatment condition.

#### Caspase 3/7 assay

For caspase assay, the same number of cells (40,000 cells/well) was seeded in 96-well plate and maintained as described above. After OGD treatment for 2 hours, caspase 3/7 assay was examined following the manufacturer's protocol (Promega, WI). Briefly, examination of caspase activity was performed by adding caspase assay solution immediately after OGD. Following incubation at room temperature, the intensities of chemiluminescence were measured and calculated following the procedures mentioned above. The intensities were compared between minocycline-treated and vehicle-treated OGD groups after subtracting the mean of no OGD control group.

#### Immunoblotting

For Western blot of Bcl-2, cultured cells were extracted and homogenized by solution containing 20 mM Tris-HCl (7.6), 150 mM NaCl, 1% NP40, 1 mM PMSF, 1 μg/ml leupeptin, 1 μg/ml TPCK and 1 μg/ml TLCK. For cytochrome c assay, cultured cells were extracted following the manufacturer's protocol (BioVision, CA). Briefly, cells were homogenized in ice-cold buffer containing protease inhibitors. After centrifugation at 700 g for 10 minutes at 4°C, the supernatant was further centrifuged at 12,000 g for 40 minutes at 4°C. Thereafter, the supernatant was collected as cytosol fraction, and the pellet was resuspended with mitochondria extraction buffer containing DTT and protease inhibitor, and stored as mitochondria fraction. Collected samples (50 μg) were loaded into 12.5% SDS-PAGE electrophoresis and transferred to a nitrocellulose membrane. After blocking by 3% skim milk in 10 mM Tris-HCl (pH 7.6), 150 mM NaCl and 0.3% TritonX at room temperature for one hour, the blot was probed with a monoclonal antibody against Bcl-2 (1:2000, Chemicon, CA), and cytochrome c (1:500, Pharmigen, CA), and visualized using a HRP-conjugated anti-mouse IgG antibody and chemiluminescence system (Amersham, UK).

#### Immunocytochemistry

Each 1 × 10^5 ^cells were plated on 8 well Permanox^® ^slides (Nalge Nunc Int, IL) at two days before fixation. Cultured cells were treated with 4% paraformaldehyde (PFA) for 10 minutes at room temperature after rinsing with phosphate buffered saline (PBS). After blocking reaction with 10% normal goat serum (Vector, CA), cells were incubated overnight at 4°C with an anti-Bcl-2 monoclonal antibody (1:100, Chemicon, CA), or anti-MAP2 polyclonal antibody (1:1000, Chemicon) with 10% normal goat serum. After several rinses in PBS, cells were incubated for 45 minutes at room temperature in FITC-conjugated anti-mouse IgG (1:1000, Molecular probe, CA), or Rhodamine-conjugated anti-rabbit IgG (1:2000, Molecular probe, CA) for visualization. Cells were processed for DAPI. immunostaining then subsequently embedded with mounting medium. Immunofluorescent images were visualized using Zeiss Axiophot 2 and the number of immunopositive cells was counted per high power field view selected at random (50,000 μm^2^). In addition, control studies included exclusion of primary antibody and substituted with 10% normal goat serum in PBS. No immunoreactivity was observed in these controls. All studies were conducted in quadruplicates, with n = 100 per treatment condition. Assessments were performed blindly by an independent investigator.

#### TUNEL staining

Cultured cells were washed with PBS. As described in our previous report [59], the TUNEL staining was carried out with DNA fragmentation detection kit (Roche, Mannheim, Germany), which detects double-strand breaks in genomic DNA with diaminobenzidine. The number of TUNEL positive cells was counted per high power field view selected at random (200,000 μm^2^) via Zeiss Axiophot 2.

### In vivo study

#### Stroke surgery

Sprague-Dawley, male 10-week old rats, weighing about 250 g, were anesthetized with gas inhalation composed of 30% oxygen (0.3 L/min) and 70% nitrous oxide (0.7 L/min) mixture. The gas was passed through an isoflurane vaporizer set to deliver 3% to 4% isoflurane during initial induction and 1.5% to 2% during surgery. Transient unilateral focal ischemia was produced using a well-established middle cerebral artery occlusion (MCAo) using the intraluminal suture model as previously described [53,60]. Physiological parameters, via blood gas assays (using the tail vein for sampling), and ischemia and reperfusion levels determined by Laser Doppler measurements, did not differ across all MCAo stroke groups. The body temperature of animals was maintained at 37°C during the surgery until they recovered from anesthesia. Based on our pilot studies, a 30-minute MCAo produces a well-delineated striatal penumbra with minimal necrotic region. Laser Doppler was used during the 30-minute occlusion period to verify reduction in blood flow, with the probe placed on the dura using rostro-caudal and lateral coordinates (AP: +2.0, ML: ± 2.0) relative to bregma. Insertion of the intraluminal filament led to 80% or greater reduction in cortical blood flow, which was used as criterion for inclusion of animals to the study and their subsequent random assignment to the treatment groups. TTC staining at 24 hours after MCAo revealed a small striatal infarct core with sparing of much of the striatum and cortex. Ischemic damage progressed beyond this time point and by 72 hours post-stroke the infarct included more striatal tissue and a substantial amount of cortex. The term "peri-infarct" is subsequently used here to refer to the tissue adjacent which became incorporated into the infarct beyond the 24-hour period. The mortality rate for the present MCAo study was 3 animals from original 33 animals, which equate to about 10%; these animals died immediately after stroke surgery. Minocycline doses of 20 mg/kg or 100 mg/kg in 5 ml saline or vehicle were administered intravenously (via the jugular vein) as a single bolus at 60 minutes after the reperfusion. This dosing regimen of minocycline was based on our previous papers [29,37].

#### Behavioral tests

Behavioral estimation was performed by using semi quantitative analysis of motor asymmetry (elevated body swing test, EBST) and neurological function (Bederson test) at 72 hours just prior to euthanasia as previously described [60-62]. The analyses of Bederson data were from raw individual scores generated from a scale of 0-3, in the order of severity of impairments. To prevent any examiner's bias, all behavioral evaluations were performed by an investigator blinded to the treatment conditions.

#### Infarct estimation via 2,3,5-triphenyltetrazolium chloride (TTC) staining

After behavioral testing at 72 hours post stroke, animals were anesthetized with a lethal dose of equithesin (500 mg/kg, i.p.), decapitated and the brains harvested. Histological determination of infarct volume was performed using standard TTC staining, and quantitative image analysis was carried out as previously described [63-65]. Infarct volume (mm^3^) was determined using the following formula = 2 mm (thickness of the section) × [sum of the infarction area in all brain section (mm^3^)]. To minimize artifacts produced by postischemic edema in the infarcted area, the infarction area in the ipsilateral hemisphere was indirectly measured by subtracting the noninfarcted area in the ipsilateral hemisphere from the total intact area of the contralateral hemisphere. However, because edema extends beyond the border of the infarct, into peri-infarct tissues, the 72-hour time point of TTC assay might have likely represented maximum edema as brain swelling caused by focal ischemia started to resolve beyond this time point. Because cell densities are based on cell counts within a defined area, the results are likely to have been influenced by edema.

### Immunohistochemistry

Under deep anesthesia, rats were sacrificed at 72 hours after reperfusion, and perfused through the ascending aorta with 200 ml of cold PBS, followed by 100 ml of 4% PFA in PBS. Brains were removed and post-fixed in the same fixative for 3 days followed by 30% sucrose in phosphate buffer (PB) for 1 week. Six series of coronal sections were cut at a thickness of 30 μm by cryostat and stored at -20°C. Free floating sections for immunohistochemistry were incubated overnight at 4°C with an anti-Bcl-2 monoclonal antibody (1:50, Chemicon), anti-MAP2 polyclonal antibody (1:500, Chemicon), or anti-GFAP polyclonal antibody (1:500, Chemicon, CA) with 10% normal goat serum. After several rinses in PBS, the sections were visualized following the method described above with modification to accelerate FITC with biotin conjugated anti-mouse IgG antibody and FITC conjugated streptoavidin (1:500, Sigma, MO). Control studies included exclusion of primary antibody substituted with 10% normal goat serum in PBS. No immunoreactivity was observed in these controls. Furthermore, TUNEL staining was performed as described in *in vitro *section, using DNA fragmentation detection kit (Roche, Mannheim, Germany). Finally, brain sections were counterstained with cresyl violet stain. Immunofluorescent and light microscopy were carried out using Zeiss Axiophot 2. Sections were blind-coded and Abercrombie's formula [66] was used to calculate the total number of immunopositive cells.

### Morphological Analysis

The density of the Bcl-2 positive cells and TUNEL positive cells in the ischemic peri-infarct area (determined by cresyl violet stain using consecutive sections) was estimated and analyzed as described previously [67]. Briefly, the level of +0.2 mm anterior to the bregma based on the atlas of Paxinos and Watson [68] was selected for semi-quantitative analysis. For estimation of TUNEL-positive cells, TUNEL positive cells were counted in four consecutive 0.05 mm^2 ^regions of the outer boundary zone of each medial striatal and cortical infarction. The total number of TUNEL positive cells with agglutinated nuclei in the four areas was counted and expressed as cells/mm^2 ^for statistical analyses. For estimation of Bcl-2 positive cells, two striatal areas (each area: 0.05 mm^2^) in the ischemic peri-infarct area and symmetrical two areas in the contralateral side were analyzed using Scion Image software (Scion Corp., MD). The areas were captured, binary images created with a distinct threshold, then the positive areas calculated and summed up. The ratio of lesion to intact side was used for statistical analyses. Additionally, confocal analysis was performed using a Zeiss LSM 510 confocal Laser scanning microscope.

### Statistics

In order to determine significant differences in cerebral infarcts, motor deficits, the number of TUNEL positive cells and Bcl-2 positive cells were analyzed using Repeated Measures of ANOVA followed by post hoc Scheffe's test. For Bederson neurological deficits, the non-parametric Kruskal-Wallis test was performed. Statistical significance was preset at p < 0.05.

## Authors' contributions

NM assisted in study conceptualization, design and coordination, and also carried out the histological and molecular assays and drafted the manuscript. TY performed the behavioral tests and immunohistochemical analyses. KH assisted in stroke surgeries and histological procedures. LX performed the stroke surgeries and assisted in histological analyses. MM assisted in the molecular assays and analyses. GY assisted in behavioral, surgical and histological assays. YK assisted in molecular analyses. KO participated in data analyses and manuscript write-up. DCH assisted in study design and manuscript write-up. CVB conceived the study, supervised its design and coordination, and led the manuscript write-up. All authors read and approved the final manuscript.
